The article "Enhancing lung cancer detection through hybrid features and machine learning hyperparameters optimization techniques" was retracted in 2025. Reasons: unreliable results or conclusions; concerns about the citations.

# Enhancing lung cancer detection through hybrid features and machine learning hyperparameters optimization techniques

**DOI:** 10.1016/j.heliyon.2024.e26192

**Published:** 2024-02-14

**Authors:** Liangyu Li, Jing Yang, Lip Yee Por, Mohammad Shahbaz Khan, Rim Hamdaoui, Lal Hussain, Zahoor Iqbal, Ionela Magdalena Rotaru, Dan Dobrotă, Moutaz Aldrdery, Abdulfattah Omar

**Affiliations:** a Center for Software Technology and Management, Faculty of Information Science and Technology, Universiti Kebangsaan Malaysia, 43600, Bangi, Selangor, Malaysia; b Health Informatics Laboratory, Cancer Research Institute, Chifeng Cancer Hospital (Second Affiliated Hospital of Chifeng University), Medical Department, Chifeng University, Chifeng City, Inner Mongolia Autonomous Region, 024000, China; c Department of Computer System and Technology, Faculty of Computer Science and Information Technology, Universiti Malaya, 50603, Kuala Lumpur, Malaysia; d Children's National Hospital, 111 Michigan Ave NW, Washington, DC, 20010, United States; e Department of Computer Science, College of Science and Human Studies Dawadmi, Shaqra University, Shaqra, Riyadh, Saudi Arabia; f Department of Computer Science and Information Technology, King Abdullah Campus Chatter Kalas, University of Azad Jammu and Kashmir, Muzaffarabad, 13100, Azad Kashmir, Pakistan; g Department of Computer Science and Information Technology, Neelum Campus, University of Azad Jammu and Kashmir, Athmuqam, 13230, Azad Kashmir, Pakistan; h School of Computer Science and Technology, Zhejiang Normal University, Jinhua, 321004, China; i Department of Industrial Engineering and Management, Lucian Blaga University of Sibiu, Bulevardul Victoriei 10, Sibiu, 550024, Romania; j Faculty of Engineering, Lucian Blaga University of Sibiu, Bulevardul Victoriei 10, Sibiu, 550024, Romania; k Department of Chemical Engineering, College of Engineering, King Khalid University, Abha, 61411, Saudi Arabia; l Department of English, College of Science & Humanities, Prince Sattam Bin Abdulaziz University, Saudi Arabia

**Keywords:** Classification, Haralick texture features, Lung cancer types, Autoencoder and gray-level co-occurrence (GLCM)

## Abstract

Machine learning offers significant potential for lung cancer detection, enabling early diagnosis and potentially improving patient outcomes. Feature extraction remains a crucial challenge in this domain. Combining the most relevant features can further enhance detection accuracy. This study employed a hybrid feature extraction approach, which integrates both Gray-level co-occurrence matrix (GLCM) with Haralick and autoencoder features with an autoencoder. These features were subsequently fed into supervised machine learning methods. Support Vector Machine (SVM) Radial Base Function (RBF) and SVM Gaussian achieved perfect performance measures, while SVM polynomial produced an accuracy of 99.89% when utilizing GLCM with an autoencoder, Haralick, and autoencoder features. SVM Gaussian achieved an accuracy of 99.56%, while SVM RBF achieved an accuracy of 99.35% when utilizing GLCM with Haralick features. These results demonstrate the potential of the proposed approach for developing improved diagnostic and prognostic lung cancer treatment planning and decision-making systems.

## 1 Introduction

Contemporary statistics on lung cancer from 2022 [1] indicate that 2.36 million new cases are expected to be diagnosed, with 85% classified as non-small cell lung cancer (NSCLC). Small cell lung cancer (SCLC) is another type of lung cancer, and both exhibit distinct treatment plans and dissemination patterns. NSCLC, characterized by slow growth, differs from SCLC, which grows rapidly and forms tumors. Lung cancer deaths are predominantly linked to cigarette smoking [2]. The term "non-small cell lung cancer" arises from the microscopic appearance of NSCLC cells, contrasting with the small, uniform cells of SCLC [3]. While smoking, radon exposure, and air pollution are common causes, NSCLC can also develop in individuals who have never smoked. Individuals experiencing any of these symptoms, particularly if persistent or worsening, should seek medical attention promptly for evaluation for NSCLC.

Small cell lung cancer (SCLC) – a rapidly growing and aggressive form – accounts for approximately 10–15% of all lung cancer diagnoses [4,5]. This distinct type, named for the microscopic appearance of its uniform, diminutive cells, primarily affects smokers but can also occur in never-smokers. SCLC's tendency to spread early to other organs often leads to advanced-stage diagnoses. Imaging tests like CT scans or chest X-rays assist in initial detection, but confirmation usually requires a biopsy. Treatment for SCLC typically combines chemotherapy and radiation therapy [6]. Surgery might be an option for isolated cases confined to specific chest areas.

Due to its aggressiveness, early diagnosis and intervention are crucial in improving SCLC outcomes. The median survival time after diagnosis, unfortunately, stands at around one year, highlighting the urgency of swift action.

Artificial intelligence (AI) is poised to dramatically reshape lung cancer detection and diagnosis [6]. One powerful approach uses AI algorithms to scan medical images like CT scans for lung cancer signatures, aiding radiologists in faster and more accurate diagnoses [7]. Beyond detection, AI can also predict disease progression and treatment response through sophisticated feature extraction techniques [[8], [9], [10], [11], [12]]. This nascent technology holds immense promise for significantly improving lung cancer care for patients. However, further research is crucial to fully unlock AI's potential and manage its limitations in this critical field.

Researchers have employed a variety of machine learning and deep learning techniques for classification and prediction tasks across diverse imaging and signal modalities. Machine learning algorithms are increasingly prominent in medical diagnostic systems, particularly for lung disease prediction. Researchers have developed standardized toolkits for feature importance calculation [13], as well as machine learning algorithms for prioritizing CT exams in emergency departments [14], and electronic noses capable of differentiating COPD patients from healthy individuals [15,16]. Liquid biopsy techniques have demonstrated promising results in lung cancer diagnosis and prognosis [17]. Additionally, blood cadmium levels have been investigated as a potential lung cancer biomarker, particularly in former smokers [18].

These advancements hold great potential for improving lung disease diagnosis and treatment. Abbasi, S. F et al. [19] used machine learning ensemble methods to accurately predict the EEG-Based Neonatal Sleep Stage. Abbasi, S. F. et al. [20] also utilized deep learning for real-time neonatal sleep stage classification. Aamir, S. et al. [21] utilized machine learning techniques for breast cancer prediction.

In machine learning, the most important and tedious task is to extract the most relevant features. In the past, researchers utilized various feature extraction approaches. Almutairi, S. et al. [22] used the gorilla troops optimization (GTO) algorithm for feature selection to detect breast cancer from a deep learning feature space. Park, H. J. et al. [23] computed the hybrid feature approach for object detection. Leng, L. et al. [24] used low correlation features for palmprint coding and verification. Leng, L. et al. [25] also utilized high discrimination-based features to detect the palmprint. Recent research [[26], [27], [28], [29], [30], [31], [32], [33], [34]] delves into a diverse toolbox of feature extraction methods, from single approaches to hybrid combinations, to analyze key cancer indicators. These tools, including texture analysis, GLCM (Gray Level Co-occurrence Matrix), and Haralick textures, along with morphological features, are then paired with powerful supervised machine learning algorithms like support vector machines, decision trees, and Bayesian classifiers. This potent combination has yielded promise.

A crucial study [35] demonstrated that low-dose spiral CT scans significantly outperform conventional chest X-rays in detecting early-stage lung cancer. While lung cancer often manifests as solitary pulmonary nodules (SPNs) on CT scans, differentiating them from benign lesions like tuberculosis or fungal infections can be challenging due to their similar appearance [36]. Enter helical CT, a game-changer introduced in 1991 that revolutionized chest imaging quality [37]. By employing multiple rows of detectors (ranging from 4 to a staggering 128), these cutting-edge scanners deliver rapid, high-resolution images of the thorax. This translates to a richer volume of information for clinicians, enabling more accurate detection and diagnosis of lung abnormalities.

Previous studies in this area often relied on basic data preparation, a single method for extracting features from images, and standard settings for their machine learning algorithms. These limitations can affect the accuracy of the analysis. While [38], explored this dataset using entropy-based complexity techniques on CT scans, their approach involved minimal preprocessing and only one feature extraction strategy. To address the dataset's imbalanced nature and small size, we implemented 10-fold cross-validation along with augmentation techniques like random cropping, flipping, and noise injection. This helps prevent overfitting, a common issue with limited data. Feature extraction plays a vital role in prediction accuracy, and researchers continuously develop new tools to improve this process. Choosing the right mix of features, single or hybrid, can significantly impact diagnostic outcomes. Think of complex diagnoses as locked doors. Different features are like keys, and hybrid approaches are like master keys that open the door more reliably than any single key alone.

The main contributions of this study can be summarized as follows:

**Combining Feature Power:** Instead of relying on a single feature type, we embraced a hybrid approach, extracting diverse features like GLCM, Haralick textures, and even those generated by an autoencoder neural network. We then "mixed" these features through concatenation, ensuring each type contributed to the analysis. As far as we know, this novel combination of hybrid features, diverse preprocessing, and optimized parameters is a first, and it significantly boosted our prediction accuracy.

**Tuning the Algorithm:** Just like fine-tuning a musical instrument, optimizing the settings (hyperparameters) of machine learning algorithms can greatly improve their performance. We used a systematic grid search technique to find the ideal settings for each algorithm. Then, we fed our single and hybrid features (again, through concatenation) into these optimized algorithms, yielding the impressive results showcased in Fig. 1. As you can see, our proposed approach takes the top spot in terms of detection performance!

**Fig. 1:** Hybrid features based a) Schematic diagram b) GLCM quantitative features from CT images.

Fig. 1a): Workflow Overview.

1. Image Input: The process begins with loading lung cancer images as input.
2. Feature Extraction: From these images, we extract crucial features of two types: those generated by an autoencoder neural network and traditional texture features like Haralick and GLCM (Fig. 1b showcases examples of GLCM features for different cancer types.).
3. Single and Hybrid Approaches: We utilize both single-feature and hybrid-feature extraction strategies. In the hybrid approach, features are combined strategically, such as GLCM + Autoencoder, Haralick + Autoencoder, or GLCM + Haralick.
4. Machine Learning Analysis: These single and hybrid features are then fed into robust machine learning classifiers like SVM with various kernels, Naive Bayes, and Decision Trees. To maximize their performance, we optimize their internal parameters.

Section one provides an introduction of the research problem background and flow of work. Section two provides Materials and methods including dataset sources, pre-processing methods, parameter optimization methods, training and testing data validation, feature extraction methods, machine learning classification methods. Section three detailed the results and discussions. Section four depicts the conclusion with summary and main findings of the study.

## 2 Materials and methods

### 2.1 Datasets

Our data comes courtesy of the Lung Cancer Alliance (LCA), who generously make it available on their website (https://wgntv.com/news/medical-watch/early-lung-cancer-detection-the-lifesaving-scan-many-smokers-skip/). This valuable resource has been used in other studies, such as [38], and comprises DICOM-format images from 76 patients with lung cancer. In total, there are 945 images, with 377 showcasing non-small cell lung cancer (NSCLC) and 568 depicting small cell lung cancer (SCLC).

### 2.2 Pre-processing

Before diving into analysis, computer vision tasks often involve image pre-processing [39,40]. Think of it as tidying up a room before welcoming guests: it enhances the image's quality, making it easier to segment, analyze, and extract key features.

#### 2.2.1 Image resize

Shrinking or stretching an image to fit a frame, save space, or sharpen details – that's image resizing [41]. We used a clever technique called interpolation, where new pixels are "guestimated" based on their neighbors, helping us resize without warping the image. But it's not just about shrinking or stretching! Keeping the "shape" of the image matters too. That's where aspect ratio, the width-to-height proportion, comes in. Ignoring it can stretch or squish the image unnaturally [42]. To avoid this, we resized proportionally, like adjusting both height and width equally, or used a built-in "keep aspect ratio" feature.

#### 2.2.2 Data augmentation

Data augmentation is a technique that artificially adds spice to your dataset by creating new versions of your existing data [43]. This helps combat overfitting, a problem where the model becomes too focused on the specific training examples and can't perform well on unseen, new data. By boosting the size and variety of the training data, data augmentation helps the model generalize better and become more reliable overall.

### 2.3 Hyperparameters optimization

Think of a machine learning algorithm like a baker preparing a cake. While the ingredients (training data) are crucial, the recipe's instructions (hyperparameters) can drastically affect the outcome [44]. These predefined settings, set before baking (training), guide the algorithm's learning process and determine its effectiveness.

### 2.4 Grid search method

Finding the sweet spot for your machine learning model is like mixing a perfect cocktail. Just as the right ratios of ingredients make a tasty drink, choosing the ideal settings (hyperparameters) can make your model perform at its best. Grid search, like a meticulous bartender trying every possible combination, systematically tests predefined hyperparameter values, picking the winner based on validation data performance [[45], [46], [47], [48]]. Random search, on the other hand, is a bit more spontaneous, throwing darts of random hyperparameter combinations and keeping the one that hits the validation bullseye. Grid search, while reliable, can become a slow and thirsty process, especially with complex models or many knobs to tweak [[45], [46], [47], [48]]. This is where swifter approaches like randomized search and Bayesian optimization come in. These techniques explore the hyperparameter space more nimbly, often reaching the peak performance point much faster than grid search.

### 2.5 Training/testing data validation

This popular technique splits the data into ten equal parts, called "folds," then trains the model on nine of them while testing it on the remaining one [49]. This process is repeated ten times, with each fold taking turns as the test set. This rigorous approach helps assess the model's general performance, not just how well it fits the specific training data [50].

### 2.6 Feature extraction

This technique identifies and extracts key features from datasets, reducing redundancy and capturing the most relevant information for analysis. Before computers can learn from data, we need to clean it up and extract the key ingredients: features! This step, called feature extraction, comes before feeding the data to the model. The objective is to identify features that hold the greatest significance for the specific task and uncover the pattern in the data. The specific feature extraction is the preliminary step in Machine learning techniques. Researchers have recently developed hybrid features [[51], [52], [53]] and explored various feature extraction methods [28,34,[53], [54], [55]] to improve the detection of different imaging pathologies. This study employs feature extraction strategies based on the GLCM, Haralick, and Autoencoder. Before feeding data to a machine learning model, we often need to "mine" for the most valuable nuggets of information.

Previously researchers [[51], [52], [53]] developed different feature extraction methods [28,34,[53], [54], [55]] for improving different pathologies in medical imaging problems. This study utilized the single and hybrid of following feature extracting approach.

#### 2.6.1 Haralick texture features

To capture the intricate textures within the images, we relied on Haralick features. These handy tools have proven their worth in classifying different types of data, like colon biopsies [56,57]. In our case, we're pioneering the use of Haralick features to analyze lung cancer patterns in CT scans.

#### 2.6.2 Gray level Co-occurrence matrix (GLCM)

GLCM is a classic texture analysis technique for a reason. This powerful tool dives deeper than just looking at pixels, exploring how they relate to each other. Think of it as analyzing not just the individual brushstrokes in a painting, but also how they come together to create the bigger picture.

The GLCM features were first proposed by Haralick. Consider an image which have $N_{x}$ column and $N_{y}$ row. Consider, gray level to quantize to $N_{g}$ levels. Let the column represented by $L_{x}=1,2,3,4,5,6\ldots \ldots \ldots .N_{x}$ and row represented by $L_{y}=1,2,3,4,5,6\ldots \ldots \ldots .N_{y}$ and set of $N_{g}$ quantized gray level denoted by $H=1,2,3,4,5,6\ldots \ldots \ldots .N_{g}$. The texture data framework is denoted by matrix of comparative frequencies $Q_{u,v}$ having two adjacent pixels parted by shift c and angle θ. The GLCM features are computed using equation (1)):

(1) $$\begin{array}{c} Q\left(u,v,d,0\right)=\{\left(x_{1},y_{1}\right),\left(x_{2},y_{2}\right)\;f\left(x_{1},y_{1}\right)=i\\ H\left(\;x_{2},y_{2}\right)=j,\left(x_{1},y_{1}\right)-\left(x_{2},y_{2}\right)=c\\ K=\left(x_{1},y_{1}\right),\left(x_{2},y_{2}\right) \end{array}$$

Here x,y denote the number of occurrences within windows magnitudes, the 1st pixel is $\left(x_{1},y_{1}\right)$ and 2nd pixel $\left(x_{2},y_{2}\right)$ denote the strength rank of derivatives from v to u. The distance between the pixel is denoted by c, the point of view between th pixel is denoted by θ. Synchronization matrix is inherently not symmetric. For GLCM to be symmetric, one of the viewpoints up to 180° required to be measured. equation (2)): is computed to formulate the symmetric synchronization matrix.

(2) Q(u,v,d,0)k=(Q(u,v,d,0)+Q(u,v,d,0),T)dividby2

Where Q(u,v,d,0),T is a transpose of Q(u,v,d,0). Possibility approximations are obtained to divide each entry in Q(u,v,d,0) by the sum of entirely probable intensity variations $\left(K_{x},K_{y}\right)$ with the space d and track θ i.e.

$$\left(K_{x},K_{y}\right),d,0$$

Thus, a normal form of GLCM is gained is computed using equation (3)).

(3) $$Q{\left(u,v,d,0\right)\;}^{X}=\frac{P\left(i,j,d,\theta \right)+P^{T}\left(i,j,d\theta \right)}{2*\sum \theta L_{x}L_{y},d,\theta }$$

Where, $Q{\left(u,v,d,0\right)\;}^{X}$ is standardized GLCM. The expression:

$${2\times (K}_{x},K_{y}),c,0$$

Equation (3) is constant, and equation (2) can be modified as in equation (4)) to be appropriate and to evade separation on the FPGA represented by equation (4)).

(4) $$Q{\left(u,v,d,0\right)\;}^{N}=\frac{P\left(i,j,d,\theta \right)+P^{T}\left(i,j,d\theta \right)}{2*\sum \theta L_{x}L_{y},d,\theta }$$

For a displacement vector d(dx,dy), the elements of a G×G GLCM are identified as Pd=(i,j)=|{((r,s)),(t,v)):I(r,s)=i,I(t,v)=j}|, where I indicate the GLCM image value and (r,s),(t,v) and (dx,dy) is the cardinality set. Let Q(u,v,d,0) is occurrence of rate. Medical imaging plots are like visual fingerprints for cancer diagnoses, helping classify and assess tumors [58].

#### 2.6.3 Autoencoder

Imagine trying to pack your entire wardrobe into a tiny suitcase without sacrificing your favourite outfits! Autoencoders, a type of artificial brain, can do something similar with data. They squeeze it down into a smaller, neater version, called a "latent space," without losing the important bits. This compressed form helps remove noise and clutter, making it easier to analyze and extract crucial features, like packing only the clothes you'll actually wear.

Autoencoder takes trajectory i=[0,1],d and first plots it to an unseen picture j=[0,1],d over a regulate plotting $j=f_{0}\left(x\right)=k\left(wx+b\right)\text{,}$ parameter by 0={w,b}. W is a d×d bulk matrix and b is a prejudice vector.

The Weight matrix w i.e. w=(wt), pre-trained weights are often beneficial when your task aligns closely with the task the weights were initially trained on. This allows for knowledge transfer and faster convergence. To abate the standard rebuilding error as reflected in equations (5), (6))):

(5) $$\theta^{*},\theta^{\prime *}=\arg_{\theta ,\theta^{\prime }}\frac{1}{n}\;\sum_{i=0}^{n}L\left(x^{\left(i\right)},z^{\left(i\right)}\right)$$

(6) $$\arg_{\theta ,\underline{\theta }}\frac{1}{n}\;\sum_{i=0}^{n}L\left(x^{\left(i\right)},g_{\theta }\left(f_{\theta }\left(x^{\left(i\right)}\right)\right)\right)$$

Corresponding likelihoods (Bernoulli's) is represented by equation 7):

(7) $$L_{H}\left(x,z\right)=H\left(B_{x}\;\|\;B_{z}\right)=-\;\sum_{k=1}^{d}x\left(x_{k}\;\log\;z_{k}+\left(1-x_{k}\right)\mathrm{Log}\;\left(1-z_{k}\right)\right)$$

If x is a binary vector, the negative log-likelihood (x, z) can be expressed. For the given example x, the Bernoulli parameters are set as z. The equation can be written as depicted in equation (8)):

(8) $${\;\theta }^{*},\theta^{\prime *}=\arg_{\theta ,\theta^{\prime }}E_{q^{o}}\left(x\right)\left[L_{H}\left(X,g_{\theta }\left(f_{\theta }\left(X\right)\right)\right)\right]$$

##### 2.6.3.1 Hybrid features

Hybrid features combine multiple types of information, like image textures and extracted data patterns, to boost a model's performance [56]. We used them by simply stitching together [57] (concatenating) different features we extracted from lung cancer images [59,60].

While hybrids can pack a punch, they can also make the model a bit more complex and demanding to run [61,62]. But the benefits often outweigh the challenges: studies show hybrid features can significantly improve accuracy in various tasks [[61], [63], [64], [65]]. In this paper, we explore three hybrid combinations: Haralick + GLCM, GLCM + Autoencoder, and Autoencoder + Haralick. Each adds a unique perspective to the puzzle, helping our model identify lung cancer nodules more effectively. We chose these specific features because no single one tells the whole story [66]. Haralick and GLCM capture image textures, while Autoencoder uncovers hidden patterns. By putting them together, we get a richer picture of the data, leading to better results. The procedure is outlined in Table 1, Table 2 regarding single and hybrid feature strategy.

**Table 1:** Single Features extraction strategy.

GLCM (22)	Haralick (14)	Autoencoder (50)
Autocorrelation	Contrast	Latent variables
Contrast	Variance	Encoder features
Correlation1	Sum Avg.	Bottleneck features
Correlation2	Sum Ent.	Reconstruction features
Cluster shade	Correlation	Decoder features
Energy	Maximal Correlation Coefficient	Other features including textures, edges, colors or shapes
Cluster Prominance	Diff. Entropy	
Homogenity2	Inf. measure of Corr1	
Sum avg	Inverse Diff. Movement	
Sum entropy	Sum Var. Entropy	
Dissimilarity	Diff. Var.	
Entropy	Info. measure of Corr2	
Inf. measure of Corr1		
Inverse Diff. Movement normalized.		
Homogenity1		
Info. measure of Corr2		
Diff. Ent.		
Inverse Diff.		
Max. Probability		
Sum of Sqr. Var.		
Sum Var.		
Diff. Var.		
Inverse Diff. Normalized

**Table 2:** Hybrid features approach.

Haralick + GLCM (36)	Autoencoder + GLCM (72)	Autoencoder + Haralick (64)
(1–22) + (23–36)	(1–22) + (23–72)	(1–14) +(15–64)

**Table 3:** Hybrid (Haralick + (GLCM) Features based detection performance and utilizing ML Algorithms to differentiate NSCLC from SCLC.

Methods	Sensitivity	Specificity	PPV	NPV	Accuracy	FPR	AUC
**Naïve Bayes (NB)**	0.9449	0.9326	0.9568	0.9146	0.9402	0.06742	0.9895
**SVM RBF**	1	0.9831	0.9895	1	0.9935	0.01685	1
**Decision Tree (DT)**	0.9858	0.9775	0.9858	0.9775	0.9826	0.02247	0.9895
**SVM Gaussian**	1	0.9888	0.9929	1	0.9956	0.01124	1
**SVM Polynomial**	0.9982	0.9972	0.9982	0.9972	0.9978	0.002809	0.9995

##### 2.6.3.2 Algorithmic steps

Step 1 Load and preprocess the images.

• Load the images into a numpy array.
• Convert the images to grayscale, if necessary.
• Normalize the pixel values of the images to the range [0, 1].

Step 2 Compute the GLCM

• Choose the offset distance and angle for the GLCM.
• Compute the GLCM for each image.

Step 3 Compute the Haralick texture features

• Compute the Haralick texture features from the GLCM. Some common features include contrast, energy, homogeneity, and correlation.

Step 4 Compute the Autoencoder features

1. Flatten each image.
2. Extract features from the flattened image using the autoencoder.

Step 5 Combine the Haralick texture features into a feature vector

• Concatenate the GLCM, Haralick texture and Autoencoder features for each image to create a feature vector.

Step 5 Machine learning model training on the feature vector

• Train the machine learning model on the feature vector to perform the desired task, such as image classification or segmentation.

### 2.7 Classification

Classification, a widely used technique [31,[67], [68], [69]]. Let's label and understand data based on predefined categories. In our case, these classifiers analyze extracted features from lung cancer images [[59], [60], [67], [68], [69], [70], [71]] to identify potential tumors. To get a well-rounded picture, we used a 10-fold cross-validation approach, essentially repeating the sorting process ten times with different training and testing sets.

### 2.8 Area under the receiver operating characteristics (ROC) curve (AUC-ROC)

AUC-ROC, a popular tool for evaluating binary classification models [72], assesses how well they can distinguish between two classes, like apples and oranges. It does this by looking at a special curve called a ROC curve.

### 2.9 Cohens kappa

Cohen's kappa is a statistical coefficient assessing the extent of agreement between multiple raters classifying categorical data. It corrects for agreement attributable to chance alone, providing a more reliable measure of true consensus. The formula for Cohen's kappa is as reflected in equation (9)):

(9) $$Kappa=\frac{\left(po-pe\right)}{1-pe}$$

where:

• po is the observed agreement between the two raters.
• pe is the expected agreement between the two raters, given that they are rating independently.
• 1 - pe is the maximum possible agreement between the two raters, given their marginal distributions.

Cohen's kappa values range from 0 to 1, with 0 indicating no agreement and 1 indicating perfect agreement. Kappa scores in the ranges 0.01–0.20, 0.21–0.40, 0.41–0.60, 0.61–0.80, and 0.81–1.00 represent slight, fair, moderate, substantial, and almost perfect agreement, respectively.

Quadratic weighted Cohen's kappa

Quadratic weighted Cohen's kappa (QWKo) is a variant of Cohen's kappa that considers the severity of disagreements. It does so by assigning greater weight to disagreements between more distant categories. The formula for QWKo is as shown in equation (10)):

(10) $$QWKo=\frac{\left(1-po\right)}{\left(1-pe\left(w\right)\right)}$$

where:

• po is the observed agreement between the two raters.
• pe(w) is the expected agreement between the two raters, given that they are rating independently and that disagreements are weighted according to a weighting matrix w.

The weighting matrix w determines the severity of disagreements between categories. For instance, a matrix with off-diagonal elements of 1 indicates equal weighting for all disagreements, while one with zeros indicates only perfect agreement counts. QWKo's sensitivity to disagreements between distant categories makes it suitable for ordered categories, like Likert scale ratings.

## 3 Results and discussions

Our goal is to boost lung cancer detection. To achieve this, we explored a treasure trove of features from lung cancer images, like textures analyzed by GLCM and Haralick, and hidden patterns uncovered by autoencoders. We then used these features, both individually and in clever combinations, as clues for machine learning models to identify both non-small cell lung carcinoma (NSCLC) and small cell lung carcinoma (SCLC). Standard metrics helped us compare their performance and pick the winning combinations.

Fig. 2(a–c) presents the lung cancer detection results using single feature extraction strategies. Haralick texture features Fig. 2a) exhibited the highest performance, achieving an accuracy of 99.89% and an AUC of 0.9984. GLCM features Fig. 2b) yielded an accuracy of 98.69% with SVM polynomial, while SIFT features Fig. 2c) attained an accuracy of 98.31% using SVM Gaussian.

**Fig. 2:** Single features based detection performance a) Haralick texture b) GLCM c) Scale Invariant Feature Transform (SIFT) to differentiate NSCLC from SCLC using machine learning techniques.

Fig. 3(a–b) depicts the AUC) for single feature extraction approach by computing Fig. 3a) GLCM and Fig. 3b) Haralick texture features.

**Fig. 3:** AUC to differentiate NSCLC from SCLC by extracting hybrid feature a) GLCM b) GLCM + Haralick.

Using GLCM and Haralick features in combination with machine learning techniques are reflected in Table 3. The SVM polynomial achieved the highest performance, reaching an accuracy of 99.78% and AUC of 0.9995.

Table 4 presents the detection performance achieved using the hybrid (GLCM + Autoencoder) feature extraction methodology and robust machine learning techniques. A 100% highest detection performance of was yielded using hybrid features (Haralick + autoencoder, GLCM + autoencoder) utilizing SVM RBF and Gaussian, as shown in Table 4, Table 5.

**Table 4:** Hybrid (Autoencoder + GLCM) features based performance detection and employing machine learning techniques to differentiate SCLC from NSCLC.

**Methods**	**Sensitivity**	**Specificity**	**PPV**	**NPV**	**Accuracy**	**FPR**	**AUC**
**Naïve Bayes**	0.9627	0.8736	0.9233	0.9367	0.9282	0.12640	0.9358
**Decision Tree**	0.9929	0.9803	0.9876	0.9887	0.9820	0.01966	0.9358
**SVM Polynomial**	1	0.9972	0.9982	1	0.9989	0.002809	0.9999
**SVM RBF**	1	1	1	1	1	0	1
**SVM Gaussian**	1	1	1	1	1	0	1

**Table 5:** Hybrid (Haralick + Autoencoder) features based performance detection and utilizing robust machine learning techniques.

Methods	Sensitivity	Specificity	PPV	NPV	Accuracy	FPR	AUC
**Naïve Bayes**	0.9556	0.8567	0.9134	0.9242	0.9173	0.14330	0.9276
**Decision Tree**	0.9929	0.9888	0.9929	0.9888	0.9913	0.01124	0.9276
**SVM Polynomial**	1	0.9972	0.9982	1	0.9989	0.002809	1
**SVM RBF**	1	1	1	1	1	0	1
**SVM Gaussian**	1	1	1	1	1	0	1

**Table 6:** Quadratic weighted Cohen's Kappa statistics.

Kappa statistics	SVM Gaussian		SVM Polynomial	
Observed agreement (po)	0.9989		0.9880	
Random agreement (pe)	0.5256		0.5271	
Agreement due to true concordance (po-pe)	0.4733		0.4609	
Maximum possible kappa, given the observed marginal frequencies	0.9977		0.9839	
Cohen's kappa	0.9977		0.9747	
Residual not random agreement (1-pe)	0.4744		0.4729	
kappa C.I. (alpha = 0.0500)	0.9932	1.0022	0.9598	0.9896
z (k/kappa error)	435.1988	p = 0.0000	128.4947	p = 0.0000
kappa error	0.0023		0.0076	
k observed as proportion of maximum possible	1.0000		0.9906	

Table 6 reflects Cohen's Kappa statistics using SVM Gaussian and SVM polynomial based on the extracted GLCM features. Using SVM Gaussian, the observed agreement (po) is 0.9989, the random agreement (pe) is 0.5256, and the agreement due to true concordance (po-pe) is 0.4733. This indicates that there is a very high level of agreement between the two raters, and that this agreement is not simply due to chance. Cohen's kappa is 0.9977, which indicates almost perfect agreement. The kappa error is 0.0023, and the kappa C.I. (alpha = 0.0500) is 0.9932–1.0022. This indicates that the observed kappa is statistically significant. The maximum possible kappa, given the observed marginal frequencies, is 0.9977. This means that the observed kappa is very close to the maximum possible kappa, which further supports the conclusion that there is a very high level of agreement between the two raters. The ratio of the observed kappa to the maximum possible kappa is 1.0000. This indicates that the observed kappa is perfect agreement. The z-score for the observed kappa is 435.1988, and the p-value is 0.0000. This indicates that the observed kappa is statistically significant at the alpha = 0.05 level.

The AUC-ROC curves for distinguishing SCLC from NSCLC using hybrid GLCM + Haralick features are presented in Fig. 4(a–e). The mean and standard deviation values of false positive rates (FPRs) and true positive rates (TPRs) were calculated for each machine learning algorithm, and linear curves were fitted to the data. The Naïve Bayes Fig. 4a) and decision tree Fig. 4b) classifiers yielded mean FPRs of 0.4652 and mean TPRs of 0.9848, with standard deviations of 0.3021 for FPR and 0.049 for TPR. The SVM Gaussian Fig. 4c), SVM RBF Fig. 4d), and SVM polynomial Fig. 4e) classifiers achieved mean FPRs of 0.3085, 0.3085, and 0.3088, respectively, and mean TPRs of 0.8087, 0.8089, and 0.8070, with standard deviations of 0.3329 for FPR and 0.3015, 0.3329 for FPR and 0.3016 for TPR, and 0.3328 for FPR and 0.3016 for TPR, respectively.

**Fig. 4:** Hybrid (Haralick + GLCM) features based AUC to differentiate NSCLC from SCLC by computing by fitting a linear curve on the AUC along with mean and standard deviation using logarithmic scales a) Naïve Bayes, b) Decision Tree, c) SVM Gaussian, d) SVM RBF, e) SVM Polynomial.

Fig. 5(a–b) presents parallel coordinate plots for visualizing high-dimensional data. These plots represent each observation in a dataset as a line connecting its values for each variable, enabling the visualization of patterns and relationships within the data. The plots utilize GLCM features extracted from MRI images of lung cancer types. The dataset includes 356 NSCLC MRI subjects and 563 SCLC MRI subjects. Blue lines represent NSCLC cases, while red lines represent SCLC cases. Solid lines indicate correctly predicted cases, while asterisks with lines indicate incorrectly detected cases. In Fig. 5a), the validation accuracy reaches 99.9%, with true positives (TP) of 355, false positives (FP) of 1, true negatives (TN) of 563, and false negatives (FN) of 0. Fig. 5b) shows the predictions using SVM Gaussian, with true positives (TP) of 347, false positives (FP) of 9, true negatives (TN) of 561, and false negatives (FN) of 2.

**Fig. 5:** Parallel Coordinate graph by extracting GLCM features from lung cancer sub-types MRI images using a) SVM Gaussian, b) SVM Polynomial.

Table 7 summarizes the findings of the current study and compares them to those of previous studies. This study aimed to enhance lung cancer detection performance in three ways: 1) refining preprocessing steps; 2) improving feature extraction strategies; 3) parameters optimization of ML algorithms.

**Table 7:** Comparison of results with previous studies.

Author	Features Used	Performance
**Teramoto et al.** [73]	1 Shape 2 Intensity	Sensitivity = 83.00%,
**Orozco et al.** [74]	1 Texture	Sensitivity = 84.00%,
**Guo et al.** [75]	1 Texture 2 Shape	Sensitivity = 94.00%,
**Messay et al.** [76]	1 Shape 2 Gradient 3 Intensity	Sensitivity = 82.00%,
**Retico et al.** [77]	1 Texture 2 Morphology	Sensitivity = 72.00%,
**Hussain et al.** [78]	RICA features and SVM	Accuracy = 99.77%
**Dandil et al.** [79]	1 Statistical 2 Shape 3 GLCM 4 Energy	Sensitivity = 97.00%, Specificity = 94.00% Accuracy = 95.00%
This study	Single features a) Haralick (SVM polynomial) b) GLCM (SVM polynomial) c) SIFT (SVM Gaussian) Hybrid features approach (GLCM + autoencoder, Haralick + Autoencoder, GLCM + Haralick) features	Single Features a) Accuracy = 99.89% b) Accuracy = 98.69% c) Accuracy = 98.39% Hybrid features approach Specificity = 100% Sensitivity = 100%, AUC = 1.00 Accuracy = 100%

Image preprocessing is like that, but for digital pictures. It's the crucial first step where we prepare images for further analysis by removing noise, adjusting brightness and contrast, and sometimes even straightening them out. Previous approaches to lung cancer detection relied on traditional feature extraction methods, which often missed crucial information. For example, Guo et al. [75] focused on texture and shape features, reaching a sensitivity of 94.0%. Sousa et al. [80] explored a broader range with gradients, histograms, and spatial features, reaching 95.0% accuracy. Messay et al. [76] combined gradients, shape, and intensity, but only achieved 82.0% sensitivity. Dandil et al. [79] took a multi-pronged approach with GLCM, shape, statistical, and energy features, reaching their highest results: 95.0% accuracy, 97.0% sensitivity, and 94.0% specificity.

We computed single and hybrid features. The Haralick yielded an accuracy of 99.89% using SVM polynomial followed by GLCM with accuracy of 98.69% and SIFT with 98.31% accuracy using single feature extracting approach. The hybrid features yielded 100% accuracy and 1.00 AUC.

## 4 Conclusion

Our recent study aimed to enhance lung cancer detection through refined preprocessing steps, optimized feature extraction strategies, and fine-tuned machine learning hyperparameters. Employing Haralick features and SVM polynomial, we achieved the highest accuracy of 99.89% among single feature extraction approaches, followed by 98.69% with GLCM features and SVM polynomial. However, the most impressive detection performance was achieved using SVM RBF with hybrid features GLCM + Autoencoder and Haralick + Autoencoder, resulting in perfect 100% sensitivity, specificity, PPV, NPV, accuracy, and AUC. The second-highest detection accuracy of 99.56% was obtained using SVM polynomial and GLCM + Haralick features, with SVM Gaussian achieving a detection accuracy of 99.35%.

Harnessing the power of diverse data: We propose a novel approach to lung cancer detection using hybrid features, combining multiple data types like scans and tissue textures. This strategy offers several advantages over single data types:

• Enhanced Patient Representation: By capturing a wider range of information,

Leveraging diverse feature sets allows the model to capture a more multifaceted portrait of patients, thereby enhancing its ability to differentiate between cancer and non-cancer. Imagine it like having a detective with multiple lines of evidence instead of just one blurry photo.

• Improved Data Quality: Hybrid features act as built-in data filters, automatically removing irrelevant or redundant information. This reduces noise and strengthens the signal, leading to a more robust and accurate machine learning model. Think of it like cleaning up a messy crime scene before starting the investigation.
• Promising Clinical Impact: The potential benefits extend beyond detection. This approach can inform decision-making, diagnosis, and even prognosis, ultimately improving patient outcomes.

Addressing Data Challenges: We were aware of the limitations of our study. The dataset was relatively small and imbalanced, which could lead to overfitting. However, we employed several strategies to mitigate this risk:

• K-fold Cross-Validation: This technique splits the data into multiple subsets, training the model on different combinations and preventing overconfidence on limited information. Imagine testing your detective skills on various cases instead of just one.
• Data Augmentation: We artificially expanded the dataset by creating variations of existing data points, providing the model with a richer training experience. Think of it like giving your detective additional evidence created from existing clues.
• Refined Preprocessing and Feature Extraction: We meticulously optimized every step of the pipeline, from data cleaning to feature selection, ensuring the model receives the most relevant and effective information. Imagine the detective honing their observation skills and focusing on the crucial details.
• Cutting-edge AI Techniques: We further enhanced prediction performance by incorporating recent advancements in artificial intelligence. Think of it as equipping your detective with the latest forensic tools.

## 5 Limitations and future directions

Further methodological improvements can be achieved through hybrid deep learning methods and optimized parameter tuning. We will also evaluate the performance using additional metrics and visualization techniques. Additionally, we will test these methodologies on larger and more diverse lung cancer datasets. Furthermore, we will incorporate clinical information alongside imaging features to enhance diagnostic accuracy and improve disease recurrence, survival, and severity predictions. The current study employed a small and imbalanced dataset and evaluated the hybrid feature extraction approach with a limited number of machine learning algorithms. Other machine learning algorithms may potentially yield even better performance. Additionally, the clinical significance of the hybrid feature extraction approach requires further evaluation. Larger datasets and comparisons with existing clinical tools for lung cancer detection are necessary. We will address these limitations by evaluating the hybrid feature extraction approach on larger and more diverse lung cancer datasets. We will also incorporate clinical information, such as patient demographics, medical history, and symptoms, to improve the performance and clinical significance of the approach. Additionally, we will compare the hybrid feature extraction approach to other state-of-the-art lung cancer detection methods. Furthermore, we will develop deep learning models capable of automatically extracting hybrid features from medical images and test the hybrid feature extraction approach for other medical imaging tasks, such as the detection of other types of cancer, neurodegenerative diseases, and cardiovascular diseases.

Finally, we will develop a hybrid feature extraction approach tailored to specific lung cancer subtypes, such as adenocarcinoma or squamous cell carcinoma, and utilize the proposed approach as a predictive model for lung cancer recurrence or survival.

## CRediT authorship contribution statement

**Liangyu Li:** Methodology, Funding acquisition, Formal analysis, Conceptualization. **Jing Yang:** Investigation. **Lip Yee Por:** Investigation, Formal analysis, Data curation, Conceptualization. **Mohammad Shahbaz Khan:** Investigation, Formal analysis, Conceptualization. **Rim Hamdaoui:** Methodology, Funding acquisition, Data curation, Conceptualization. **Lal Hussain:** Writing – review & editing, Writing – original draft, Visualization, Validation, Supervision, Software, Resources, Project administration, Methodology, Investigation, Formal analysis, Data curation, Conceptualization. **Zahoor Iqbal:** Project administration, Methodology, Investigation, Conceptualization. **Ionela Magdalena Rotaru:** Writing – review & editing, Supervision, Formal analysis. **Dan Dobrotă:** Writing – review & editing, Funding acquisition, Formal analysis. **Moutaz Aldrdery:** Writing – review & editing, Investigation, Formal analysis. **Abdulfattah Omar:** Software, Methodology, Investigation.

## Declaration of competing interest

The authors declare that they have no known competing financial interests or personal relationships that could have appeared to influence the work reported in this paper.
